The article "Analysis of e-Mail Spam Detection Using a Novel Machine Learning-Based Hybrid Bagging Technique" was published in 2022. Journal: Comput Intell Neurosci.

# Analysis of e-Mail Spam Detection Using a Novel Machine Learning-Based Hybrid Bagging Technique

**DOI:** 10.1155/2022/2500772

**Published:** 2022-08-09

**Authors:** Alanazi Rayan

**Affiliations:** Department of Computer Science, Jouf University, Sakaka, Saudi Arabia

## Abstract

e-mail service providers and consumers find it challenging to distinguish between spam and nonspam e-mails. The purpose of spammers is to spread false information by sending annoying messages that catch the attention of the public. Various spam identification techniques have been suggested and evaluated in the past, but the results show that the more research in this regard is required to enhance accuracy and to reduce training time and error rate. Thus, this research proposes a novel machine learning-based hybrid bagging method for e-mail spam identification by combining two machine learning methods: random forest and J48 (decision tree). The proposed framework categorizes the e-mail into ham and spam. The database is split into multiple sets and provided as input to each method in this procedure. Moreover, tokenization, stemming, and stop word removal are performed in the preprocessing stage. Further, correlation feature selection (CFS) is employed in this research to select the required features from the preprocessed data. The effectiveness of the presented method is evaluated in terms of true-negative rates, accuracy, recall, precision, false-positive rate, *f*-measure, and false-negative rate; the outcomes of three studies are compared. According to the results, the presented hybrid bagged model-based SMD technology achieved 98 percent accuracy.

## 1. Introduction

Over the years, e-mail has proven to be an immensely important method of communication, offering near-instant access to anyone around the world with an Internet connection. According to Tschabitscher, there was about 5 billion monthly active e-mail account in 2017, with that number likely to rise to over 5.5 billion per month in 2019. The investigator also points out that, even though over 270 billion e-mails are being sent every day, around 57 percent of them are trash. To detect spam or phishing e-mails, there seem to be several emerging machine learning algorithms and also strategies that closely match immune defense mechanisms, but overall effectiveness has been a big worry. The majority of the strategies are effective in preventing spam, but they also prevent certain nonspam communications, known as ham. This is an issue since it may result in the users losing pertinent data. Diverse kinds of e-mail assaults, including phishing, e-mail spoofing, and variations of spam e-mails, such as a covert redirect, clone phishing, spear phishing, and whaling, are continually bombarding customers worldwide. To make the warning message get sent from a valid user, e-mail spoofing frequently entails faking the e-mail header (the from portion). Spammers use mail impersonating since individuals are more likely to read an e-mail if it appears to be from someone they know [1].

Spamming, which would be described as the practice of delivering unwanted communications to a large group of people, is on the rise right now. Since reputational risk and economical disruptions are one of the spammers' highest significant things, the spam influx has prompted academia scholars to investigate this issue as a promising proposed study. As a result, both organizations and people require effective and trustworthy junk e-mail filtration solutions. To respond to the growing volume of unwanted e-mails, these computers must apply sophisticated tactics. For a long period, spam e-mail identification has indeed been intensively researched [2]. There are two types of spam e-mail filtering techniques now available: unimodal and multimodal. Message and image-based are the two categories of the first group. The earlier was established to identify spam e-mails that simply contained information, whereas the latter was designed to handle embedding textual inside graphics, understanding that fraudsters used it to bypass message solutions. Multimodal technologies, the subordinate group, are required to identify spam e-mails that contain either text or images, sometimes known as hybrid spam e-mails. Considering the number of data contained, hybrid spam e-mail seems to be more dangerous and sophisticated than image-based and message-spam e-mail. This makes it an essential process. As a result, effective methods for processing both text and visual material are required for hybrid spam e-mail. The goal of the multifunctional system is to produce relevant features using visual and textual modes before integrating these at the characteristic or choice levels [3].

Many e-mail providers have included an automated trash detection performance based on the previous e-mail transmitted records as the premise of classification. Nevertheless, there are still e-mail servers, especially those run by individuals, that do not have trash detection performance. This is because not all private e-mail products include phishing identification as one of their application software packages by the standard. As a result, a spam detection mechanism should be developed and implemented as a software program or an add-on component. However, owing to the inherent flexibility of unsolicited messages by use of mail systems, the efficacy of trash identifying systems has frequently been restricted, or in some cases made useless or corrupted, necessitating the development of stronger spam identification techniques [4]. Many spam identifying techniques have indeed been suggested and evaluated in the research; however, the claimed accuracy nevertheless calls for more research in this area to improve accuracy. Researchers used an artificial neural network-based model to identify spamming but only managed to achieve an efficiency of 86 percent, which is still far from optimal. The researchers utilized a naïve Bayes strategy for extracting features while combining expense multi-objective genetic programming for phishing detection, with an efficiency of 79.4 percent properly detecting e-mail kinds. Furthermore, the paper developed a spam identification structure based on interval derivative fuzzy sets, investigating the potential of type-2 fuzzy logic, and was only able to achieve a spam prediction performance of 86.8% for the test dataset [5].

Individuals and businesses gain greatly from the advancement of technological advancement. Simultaneously, technological advancement acts as a conduit for illicit activity. While hacker or virus utilization is a specialized talent that necessitates behaviors that are not performed by the average individual, social engineering is not as technically demanding. As a result, social engineering is becoming increasingly prevalent. In the third period of 2019, social engineering attacks have been the most common hazard to individuals and the second most common threat to businesses [6]. In most situations, media manipulation is the first stage in the progression of cybercriminals. “Cyberattacks of a network of an organization began in 81 percent of the cases with a phishing message.” A malicious program is a form of harassment that aims to steal private and personal data out of its potential victims. Phishing attacks involve a range of different methods, the much more popular of which include e-mail postings, phone conversations, social networking site messaging, and many others [7]. To combat phishing and minimize the primary cybercrime, it is critical to recognize phishing e-mails. While technological anti-phishing measures are insufficient, personal and organizational security is based on education and knowledge of the misleading assault environment. Researchers will concentrate on e-mail-based phishing assaults in this article. e-mail communications are utilized as an interactive setting to gather customized content in e-mail-based phishing scams [8].

Every day, people are inundated with hundreds of commercials. Users know how to avoid and decrease their access to information and messages that are uninteresting or unreliable throughout the term. Personal factors are one technique for advertisers to pique the interest of the customer base [9]. Marketers employ Internet shopping data to increase the relevancy of advertising and distribute them to particular customers to make companies stick out now to customers in an electronic medium bombarded with the ever-growing congestion of adverts. Personalized advertising is a paid communication “matched to a user's attributes, hobbies, or preferences.” Because tailored information is recognized being a persuasive communication tactic that favorably affects attentiveness, mental reactions, and perceptions toward advertising, the capacity to gather customer information Internet is critical [10]. Customization is intended to produce favorable responses because consumers demand to advertise that are pertinent to them, but nonrelated SNS commercials are likely ignored because they are viewed as intrusive or aggressive. As a result, prior research demonstrates this need for customization in the digital world because it enhances marketing effectiveness by making adverts more unforgettable and personable, ramping up inspiration to handle advertising messages, instituting behavior changes, and ramping up the marketing rate of response [11].

Another benefit of marketing comes from the ability to identify a particular targeted audience due to self-characteristics such as age and sexuality available on profile pages. Nevertheless, there is little study on personalized social media ads, and future studies should go beyond statistics to include information specific to social media. Conventional systems for gathering customer data may provide marketers with limited or erroneous data about customers. Because social media profiles are based on voluntary self-disclosure of private details, there is the potential for purposeful distortion, allowing for the creation of fake accounts, online trolls, and chatbots. As a result, aggregating SNS information may result in mistakes in customer profiles and focused marketing [12]. The following are the particular research materials for message spam filtering: research employs the classification tree approach to filter trash, which selects text characteristics using the RLM perceptions rather than the data gain technique. The reliability and memory rates of this technique are both over 89 percent, according to the trial data. To acquire multiple classification likelihood functions of an e-mail as junk, the study employed numerous strong classifiers, each of which uses a logarithmic regress approach to achieve the categorization confidence interval. Finally, a promoting approach is used to aggregate the several categorization likelihood functions to obtain actual data for the e-mails as junk, which will then be matched to a benchmark to evaluate whether or not the e-mail is malware [13].

Section 2 explains previous research related to this research, and Section 3 describes the methodology of our work.  Section 4 introduces to the basics of decision tree algorithms random forest and J4.  Section 5 explains the system design.  Section 6 reports on computational studies of the proposed approach, and Section 7 concludes with findings and work to be done in the future.

## 2. Related Works

Their daily lives are becoming increasingly reliant on social media. Our communication through these platforms has only grown in tandem with their fast expansion. Twitter is among the most widely used social media platforms in the Middle East. Tweet, like other social networking sites, is susceptible to spam profiles that distribute part of the strategy. Leading to a shortage of appropriate technology that serves the Arabic language, Arab countries have been among the most attacked. Furthermore, because Arabic is a sophisticated language with multiple varieties and significant grammatical rules, retrieving text data might be difficult. Several recent researches have looked into inventive ways to reduce spamming in tweets. The research collected Arabic datasets appropriate for junk identification to tackle the problem of identifying spamming identities in Arab on tweet. Utilizing Twitter's subscription application programming interface, the database included information from premium content. Abandoned identities were flagged, and information was labeled. A hybrid approach that is based on deep learning algorithms was developed, which has numerous benefits, along with more efficient and timely outcomes while using fewer system resources. Text-based statistical analyses were performed using a convolution neural network (CNN) approach, while information was analyzed using a basic neural network-based framework. When the two algorithms' outputs were pooled, they categorized identities as spam or not spam. The suggested approach surpassed the best designs evaluated thus far in the research, achieving an efficiency of 94.28 percent with the hybrid algorithm employing superior extracted features. In interaction via social media platforms like Twitter, several Arabic accents and informal idioms intersect. This makes it more difficult to identify spam identities utilizing solely text-based characteristics and therefore necessitates several earlier processes to acquire correct categorization. Additional research into a preprocessing stage that might accommodate Arabic accents with minimum impact on intentions and interpretation would have been beneficial. This is considered the major limitation of spam accounts combined with the text and meta-based deep learning framework proposed by [14].

In numerous businesses, especially marketing, the categorization, and suggestion method for recognizing social networking site (SNS) members' preferences play an important part. Customized adverts help firms stick in a sea of digital advertising by increasing relevancy to customers and eliciting positive reactions [15]. The comprehensive evaluation of photos and messages on client postings could more accurately forecast a user's preferences, even though almost all user preference categorization research had concentrated on text information. As a result, this study uses both language and visuals to classify SNS participants' preferences. The Curlie directory was used to describe the interests of consumers, and researchers compared alternative convolutional neural network (CNN) and recurrent neural network (RNN)-based models for the user preference categorization systems [16]. Convolutional neural classification methods have been used to categorize photos via individuals' SNS posts, whereas RNN-based classification methods were utilized to classify text information in their hybrid neural net system. The categorization of users' preferences fared best while utilizing text and graphics combined, at 96.5 percent, vs texts alone, 41.39 percent, or photos only, 93.2 percent, according to the findings of the thorough trials. Our suggested approach helps marketers make (1) interest-based suggestions, (2) ranked-order suggestions, and (3) real-time suggestions by giving insight into tailored SNS marketing communications. To their understanding, this is one of the earliest articles to leverage combined image and message statistics using user-generated material to enhance the effectiveness of reliably identifying the political inclinations of SNS users for such aim of improving targeted advertising experiences [17].

Single-modal spam filtering algorithms have obtained a maximum classification performance for picture and text junk in the latest days. To remain undetected by single-modal spamming filtering techniques, fraudsters introduce garbage data into the multi-modality component of an e-mail and blend it to lower the single-modal spam detection processor architectures' classification performance, so achieving the goal of dodging identification. In light of this, the latest product known as multimodal design obtained from the numerical fusing (MMA-MF) has been presented, which employs a multimodal fusing strategy to ensure that trash can be efficiently filtered whether it has been concealed in word or phrase. To filter trash, the approach integrates a convolutional neural network (CNN) with a long short-term memory (LSTM) framework. The visual and textual components of an e-mail were processed individually to use the long short-term and convolutional neural network models to generate two categorizations posterior distribution, which are then merged into a hybrid framework to estimate if the message is trash or otherwise. Researchers are using a grid search optimization algorithm to determine the most appropriate hyper-parameters for the MMA-MF designer's hyper-parameters and a k-fold cross-validation technique to assess the effectiveness of the algorithm. The findings of the experiments reveal that this approach outperforms typical spam detection algorithms, with accuracies ranging from 92.65 to 98.49 percent. Researchers believe using the novel methodology, as well as the one-class classification algorithm and the few-shot pedagogical practices, to address the problem of the discrepancy between the number of spam and nonspam e-mails, and we will keep collecting extra realistic combined electronic mail data sources to enhance the system framework of the prototype so that it could function better at phishing detection [18].

Spam e-mail makes it difficult for users of e-mail accounts to receive critical data. e-mail spam prevention has indeed been implemented in public mail servers using a variety of ways. However, not all e-mail systems offer to spam e-mail significant findings for the usage of a limited amount of enterprise e-mail addresses. To safeguard e-mail users from junk, the system administrator should implement a distinct or module junk mail detection rate. The goal of this research is to find the most effective strategy for identifying spam e-mails. To determine the most effective technique for identifying spam e-mail, researchers used machine learning techniques such as decision tree, logistic regression, and random forest, and evaluated the findings. The speed of train and test procedures, and the reliability of spam message detection are used to determine effectiveness. According to the findings of this investigation, the random forest approach has an outstanding outcome, with a testing data velocity of 0.19 seconds and a 98 percent reliability. This finding could be utilized as a basis for the formulation of various algorithms for spam filtering. The limitation of the research is the researcher assumed that more specific algorithms, like the approximate solution and the database process, would be used to enhance efficiency [19].

Smart objects supply the preponderance of computational services near to the end customers for the next-generation Internet of things. These gadgets with built-in knowledge may make autonomous choices in the context where they are placed by applying diverse AI methodologies. In response to these challenges, researchers propose a cognitive incursion prevention mechanism that prevents brand loyalty is important from infiltrating the web address bar image data, hence maintaining the legitimacy of search engine result pages. By addressing three separate levels, namely, data collecting services, edge computing services, and cloud services, the proposed model provides ambient knowledge for web data filtering and identifies web spam. The goal is to identify harmful images. The average, image gradient, and volatility of a picture are first retrieved, and afterward, the received information is analyzed in the proposed framework. For the performance evaluation of the proposed method, deep learning techniques are being used. It achieved a 98.77 percent accuracy when tested on a real-time available dataset [1].

## 3. Methodology

The e-mail is classified by the classification model based on its content and other criteria. The procedure of feature extraction and selection is critical for the majority of classification issues. In the categorization process, characteristics are quite important. The correlation-oriented feature extraction (CFS) approach is utilized for features extracted in this research [20]. For effective classification performance, the CFS technique is used to extract the best characteristics from a collection of characteristics. In the suggested spam mail detection (SMD) method, a unique hybrid bagged method is provided to address the shortcomings of the current approach. The basic mechanism of e-mail classification is depicted in Figure 1.

The suggested spam mail identification structure is predicated on the machine learning approach's efficiency. Firstly, electronic mail information is gathered through a spam mail identifying scheme. The e-mail information gathered is unorganized and unfiltered. e-mail information must be preprocessed in terms of reducing operations and providing an exact outcome. To obtainnecessary information, the information is automatically by eliminating text content, stemmed, and term text categorization. Each categorization technique uses the database, which is arbitrarily partitioned into multiple sets. To assess the ultimate classifier performance, the bagging method integrates the categorization performance of the different machine learning techniques [21].

## 4. Preliminaries

The basics of the random forest and J48 decision tree algorithms are explained in this part.

### 4.1. Random Forest

The random forest technique implements bagging by building each tree in an ensemble of decision trees from the bootstrap sampling of data from the training dataset. The length of each random subset of texts is determined by repeating randomized systematic sampling till its bootstrapping sample equals the size of the image training dataset. Just a random selection number of features is examined while creating each decision component for each decision tree [22]. The yes/no criterion that effectively lowers the unpredictability of the information is chosen for the next node in the tree from the “*k*” randomly picked attributes to examine for creating each decision point and mentioned in

(1) $$\begin{array}{c} \text{Entropy}≔=\text{pro}\left(\text{Spam}\right){\text{log}}_{2}\text{pro}\left(\text{Spam}\right)-\text{pro}\left(\text{Not Spam}\right){\text{log}}_{2}\text{pro}\left(\text{Not Spam}\right). \end{array}$$

Whenever the classification is undecided as to whether a text is a junk, the unpredictability is highest. Here is an instance of a simple spam detection random model mentioned in Algorithm 1.

Unlike many other decision tree optimization models, the random forest algorithm dataset is divided set iteratively when it is no longer effective to minimize the randomness of each leaf node (whether if all the model learns texts for a binary tree have the same categorization but because it is not able to successfully detach the spam e-mails from the nonspam texts). To use a voting approach, the full ensembles of decision nodes are then utilized to classify fresh communications [23].

Random forest is a higher-level variation of CART that uses the bootstrap bagging approach and random feature selection. In this approach, a forest is created from a large number of trees, which are subsequently analyzed to produce categorization input data [24]. The outcome consensus for each classification stage determines the outcome of categorization evaluation inputs, as shown in Figure 2.

### 4.2. Decision Tree

The J48 classification is predicated on the notion of probability and is a decision tree classification. It is a multiclass classifier that uses the training knowledge to generate decision trees. For the categorization of the new data element, the decision tree built utilizing J48 is based on the training examples feature values. J48 is based on the idea that dividing data into numerous sets allows any feature characteristic to be utilized to generate a decision [25]. The method performs in a nonlinear manner until every information characteristic is analyzed and classified; i.e., the characteristics retrieved using this method are the greatest feasible characteristics for the data category in question. The following are among some of the factors that the system takes into account:

- The technique creates judgment nodes higher in the tree whenever examples of originally thought unsupervised classification are detected
- When the data collected correspond to a single class, the algorithm is used to generate a prediction model with a leaf node and requests that category be considered
- If the characteristics or obtained features do not give any mutual information, a judgment node is generated just above the current tree using predicted values

The root of the tree, internal nodes, and leaf nodes make up a tree structure. Leaf nodes indicate the class, while nodes in the network indicate the constraints attached to characteristics and traits [26]. A sample decision tree is shown in Figure 3. For the J48 decision tree algorithm, Algorithm 2 is provided.

DT is the collection of training examples in Algorithm 2, and *F* is the decision tree. Splitting requirement is an attribute selection strategy in this method that divides the data objects into certain individual courses.

## 5. System Design

Figure 4 depicts a spam e-mail test method that employs machine learning. The first phase is data preparation, which includes data analysis and splitting. This approach sought to segregate half of the data into three categories: data training spam, data training nonspam (ham), and data testing. The data filtering process is the following step, which removes any extraneous words and expressions [27]. The investigator then constructed a model to reflect each technique that was discovered. The procedure of training and modeling testing, which has resulted in the acquisition of accuracy levels from spam e-mail classification, is the final phase. Aside from the accuracy number, another comparative criterion is the speed of the training phase when utilizing an existent database [28].

### 5.1. Framework of Spam Identification

The process of the spam mail detection (SMD) program for classifying e-mail into ham and spam messages is depicted in this part. The SMD network is comprised of strong division capabilities that were first established with the hybrid bagged method concept. The feature identification is executed using a correlation-based feature selection technique, and the analysis is performed using a unique hybrid bagging methodology [29].

The bagging strategy is a hybrid method in which the categorization aim is served by a decision tree-based J48 algorithm and random forest.  Figure 5 shows the flowchart of the SMD system for text categorization. The SMD model divides the e-mails into two categories: spam and ham e-mails [30]. The text-based e-mail database is preprocessed to allow for effective extracting features. A hybrid bagged categorization strategy is being explored. e-mail datasheet preparation, preprocessing of information, selection of features, and hybrid bagged technique are the four modules of the SMD method. In the sub-section, a working prototype was also presented [31].

### 5.2. e-Mail Dataset

The database e-mail spamming code project machine learning and AI assert were primarily seen as the information training and testing data in this study. This database is provided to competition competitors as a reference for effectively detecting spam e-mails. Information is then classified as trash or nonspam intended to assist in the detection and verification of results using machine learning methods. Again, for the spam mail detection technique, an e-mail database is created [11]. From the Ling Spam database, various messages are chosen at random. For supervised classification, the database comprises a collection of 1000 e-mails, including both ham and spam e-mail messages. The database is separated into sets for each classification method because the organization procedure is a bagged technique. A total of two pairs of 500 e-mails have been generated. Each one of the random forest and decision tree algorithms uses 300 e-mails for training and 200 e-mails for testing.  Table 1 displays the dataset's statistics.

### 5.3. Preprocessing

The message database under consideration is unprocessed. As a result, it must be preprocessed until being considered anymore. There are 3 phases in the preprocessing stage. The tokenization of the text information is measured first. Tokens are words that are separated from the rest of the phrase. Stop words are eliminated from the tokenized phrases. Inappropriate phrases with no linguistic meaning are known as stop words. During preprocessing, a document with around 670 stop words is routinely generated, and words are eliminated from the content. Stemming is the third stage in the preprocessing component. The stemming method removes a word from its root word. Stop word removal and stemming are key preprocessing processes since they significantly decrease the search area for effective extracting features [26].

### 5.4. Feature Selection

Feature selection is an important concern that has sparked a bit more articles. That has three objectives: (i) improving classification predictive performance, (ii) developing a better and more cost classifier, and (iii) gaining a greater understanding of fundamental processes related to information production. Two recommended strategies for reducing the feature set size are dimensionality reduction and relevant feature selection. Although relevant feature selection entails extracting a subset characteristic, image compression entails combining the original features and functionality linearly [32]. In every categorization system, features are quite significant. The SMD approach is based on the notion that spam mail contains different information than ham e-mail. The feature collection includes numerical keywords, languages, grammar or typographical problems, improper terms (words connected to product/service advertisements, dating, adult phrases, and so on), recurrence number, and document size, among other things. Correlation feature selection (CFS) is employed in the SMD technology. CFS simply selects the best characteristics from a range of options for increasing the overall system efficiency. “Good feature selections comprise characteristics correlated significantly with the categorization, but uncorrelated to one another,” according to the correlation-based feature selection technique.

Text data with extracted features are primarily thought of as a bag of visuals. The term frequency technique is used to display the total number of terms in a material. All phrases are counted for recurrence, and those with a recurrence under a certain level are removed. The plan proves the words' utility while concurrently dipping the search area [33]. Utilizing a correlation-based feature selection strategy, the acquired set of features is even further decreased. The correlation-based feature selection approach chooses only the feature set that is most closely connected to the given class. Equation (2) offers the system of linear equations of the correlations-driven feature selection technique if *c* is the feature set with *n* number of features and a is the set of training.

(2) $$\begin{array}{c} \text{Correlation feature selection}={\text{max}}_{s_{n}}\left[\frac{r_{ac_{1}},r_{ac_{2}},r_{ac_{3}}\ldots r_{ac_{n}}}{\sqrt{n+2\left(r_{c_{1}c_{2}}+\ldots r_{c_{i}c_{j}}+\ldots r_{c_{n}c_{1}}\;\right)}}\right]. \end{array}$$

Here, the average correlation feature class is denoted as *r*_*ac*_ and the average correlation feature-feature is denoted as *r*_*cc*_.

### 5.5. Hybrid Bagging Technique

The classification design is the fourth and final system. For categorization, a hybrid bagged technique combining the decision tree-based J48 algorithm with the random forest is being examined. The bagged strategy, also known as the bootstrapping aggregating method, reduces variability by combining numerous repeating subsets of the same database. Multiple models have been created in this method by arbitrarily partitioning the e-mail database into two independent sample mail data sources: SD1 and SD2. Separate classifiers are trained using each instance of e-mail collection. The outcome of the entire process is the average of two categorization systems' results. For multiclass recognition and classification, the J48 method and random forest are utilized [34]. The mean of the anticipated values is used to determine the classiﬁcation accuracy and the idea of bagging as depicted in Figure 6.

### 5.6. Working Process

Only with the assistance of the accompanying instance, a complete explanation of the components of the spam mail detection (SMD) process is achieved [35]. An instance of a randomized mail is used to demonstrate the spam mail identification program's step-by-step operation. As illustrated in Table 2, the SMD form includes an e-mail as input and provides spam or ham as an outcome.

## 6. Results and Discussion

The obtained measurements of the spam mail detection (SMD) method are mentioned in this report. For the experiments, an e-mail database of 1000 e-mails is used, including 500 e-mails in each of the two classification methods [36]. Three tests were carried out in all, and the findings are evaluated. Two studies employing separate random forest classification algorithms, J48 decision tree algorithms, and a third investigation utilizing a hybrid bagged technique is done for spam e-mail identification. The RF method is a straightforward supervised learning technique that is simple to comprehend and execute. Even with an insignificant number of training trials, the method generates good results. However, the technique is based on the premise that the database contains separate class features. On either side decision, the tree-based method can deal with feature relationships, incomplete information, as well as other issues. However, decision tree algorithms struggle with data stream sets and the over-fitting problem. The finest of both methods were combined in the hybrid bagged technique of random forest and the J48 method [32].

The overall outcome of a spam mail recognition model is the combination of both models' forecasts, resulting in a system that is efficient and dependable. The efficiency characteristics are used to assess the effectiveness of the implemented method spam mail detection technique. To analyze the efficiency of the spam mail detection technique, measures such as accuracy, false-positive rate, recall, precision, true-negative rate, *F*-measure, and false-negative rate are computed. The effectiveness of the spam mail detection system is assessed using the criteria listed in Table 3.

The algorithm received an average accuracy of 95 percent, which is the average of the two classification systems' efficiency. Random forest classifier has an accuracy of 84 percent, with precision and recall values of 86 percent and 82 percent, correspondingly. The J48 method, on the other hand, achieves 92 percent accuracy, with precision and recall values of 94 percent and 90 percent, correspondingly. The assessed outcomes of the three trials are presented in Table 4: random forest, J48 algorithm, and hybrid bagged technique, correspondingly. The graphical representation of Table 4 is presented in Figure 7, in which the graph is plotted for the analysis outcome of spam detection for three algorithms. The blue bar represents accuracy rate, orange bar represents the precision, gray represents the recall value, and the yellow bar represents the *F*-score.

Table 5 and Figure 8 show the comparative analysis of the true-positive (blue bar) and true-negative (gray bar) as well as the false-positive (orange bar) and false-negative (yellow bar) cases for the three algorithms. Based on the graph, it is verified that the true-positive case and the true-negative case have more performance than the others. Owing to this, Table 6 and Figure 9 show the comparative analysis of true-positive rate (blue bar), false-positive rate (orange bar), and false-negative rate (gray bar).

By comparing the J48 decision tree method to the random forest and the hybrid bagged method, the findings in Tables 4–6 clearly show that the J48 decision tree algorithm achieves higher outcomes of precision, recall, and accuracy. Nevertheless, in the instance of random forest (90 percent), the proportion value of the F-measure is larger than that in either J48 (85 percent) or the hybrid bagged technique (90 percent) (88 percent). The graphical depiction of the contrast of the SMD state's outcome and the related classification methods independently is shown in Figures 7–9.

## 7. Conclusion

Today, spammers are among the most demanding and unpleasant issues related to communication and information technologies. Paid trolls abuse this communications device by sending spam e-mails, which has a negative impact on productions and numerous Internet consumers. This research presents a spam mail detection mechanism that uses a hybrid bagging technique for execution. Random forest and decision tree (J48) are the categorization techniques employed in this technique. The hybrid bagging method-based spam mail detection system attained an overall rate of 95 percent, indicating that the testing findings are superior when using simply the J48 method. The idea of enhancing technique could have been used for future studies to improve the system's effectiveness. The enhancing strategy substitutes the weak classifier's learning features with those of the classification model, enhancing overall design competence. In future consideration, the researcher assumed that even more sophisticated techniques, like the evolutionary algorithm and the dataset procedure, will be more widely used to enhance effectiveness.

## Figures and Tables

**Figure 1:** Common e-mail filter procedure.

**Figure 2:** Mechanism process of RF.

**Figure 3:** Decision tree structure.

**Figure 4:** System design.

**Figure 5:** e-mail classification based on spam mail identification.

**Figure 6:** Bagging approach.

**Figure 7:** SMD parameter outcome on accuracy, precision, recall, and *F*-score.

**Figure 8:** Analysis outcome of true and false positive and negative.

**Figure 9:** Analysis outcome of *TN*_*R*_, *FN*_*R*_,  and *FP*_*R*_.

**Algorithm 1:** Spam detection random model algorithm.

**Algorithm 2:** Decision tree algorithm.

**Table 1:** Mail database.

Database	Random forest	Decision tree
Training ham mails	180	120
Training spam mails	130	170
Testing ham mails	150	50
Testing spam mails	110	90
Average mails	500	500
Overall	1000	

**Table 2:** Working process.

Parameter	Example
I/P	Subject: A new way to shop! Get newpass free for a year & enjoy benefits across brands! Continue to earn a minimum 5% Newcoins! Terms and conditions applied. Click here for more detail
Tokenization	“Subject” “:” “A” “new” “way” “to” “shop” “!” “Get” “newpass” “free” “for” “a” “year” “&” “enjoy” “benefits” “across” “brands” “!” “Continue” “to” “earn” “minimum” “5%” “Newcoins” “!” “Terms” “and” “condition” “applied” “.” “Click” “here” “for” “more” “detail”
Stop word elimination	“new” “way” “shop” “Get” “newpass” “free” “year” “enjoy” “benefits” “across” “brands” “Continue” “earn” “minimum” “5%” “Newcoins” “Terms” “condition” “applied” “.” “Click” “here” “more” “detail”
Stemming	“new” “way” “shop” “Get” “newpass” “free” “year” “enjoy” “benefits” “across” “brands” “Continue” “earn” “minimum” “5%” “Newcoins” “Terms” “condition” “applied” “.” “Click” “here” “more” “detail”
Outcome	Spam mail

**Table 3:** SMD evaluation measure.

Assessment parameter	Specification	Model
Precision	The efficacy of the classifier is defined by precision	*T*_*P*_/*T*_*P*_+*F*_*P*_
Accuracy	The proportion of positive forecasted value to the overall set	*T*_*P*_+*T*_*N*_/*T*_*P*_+*F*_*P*_+*T*_*N*_+*F*_*N*_
Recall	The positively labeled information provided by the classification out of the entire data	*T*_*P*_/*T*_*P*_+*F*_*N*_
*F*-score	Overall quality is demonstrated by the classifier's ability to produce efficient beneficial results.	2 × *P*.*R*/*P*+*R*
True-negative rate (*TN*_*R*_)	Spam mails managed to identify as a percentage of all spam mails.	*T*_*N*_/*T*_*N*_+*F*_*P*_
False-negative rate (*FN*_*R*_)	It detects the number of spam e-mails that have been missed.	*F*_*N*_/*F*_*N*_+*T*_*P*_
False-positive rate (*FP*_*R*_)	The number of spam e-mails mistakenly detected as a proportion of overall spam mails	*F*_*P*_/*F*_*P*_+*T*_*N*_
True positive (*T*_*P*_)	The sum of ham electronic mails that were accurately detected.	—
False negative (*F*_*N*_)	The sum of ham mails that have been mistakenly classified as spam.	—
False positive (*F*_*P*_)	The sum of spam messages that were mistakenly recognized as ham.	
True negative (*T*_*N*_)	The sum of spam e-mails that were appropriately detected.-	—

**Table 4:** Analysis outcome (1).

Parameter	Random forest	Decision tree	Hybrid bagging
Accuracy	84	92	88
Precision	85	94	90
Recall	82	90	86
*F*-score	90	85	88

**Table 5:** Analysis outcome (2).

Parameter	Random forest	Decision tree	Hybrid bagging
True positive	82	90	86
False positive	15	5	11
True negative	87	93	84
False negative	20	10	14

**Table 6:** Analysis outcome (3).

Parameter	Random forest	Decision tree	Hybrid bagging
True-positive rate	87	95	89
False-positive rate	20	10	16
False-negative rate	15	5	12

## Data Availability

The data that support the findings of this study are available from the corresponding author upon reasonable request.
